# Application of Leg, Vertical, and Joint Stiffness in Running Performance: A Literature Overview

**DOI:** 10.1155/2021/9914278

**Published:** 2021-10-21

**Authors:** Artur Struzik, Kiros Karamanidis, Anna Lorimer, Justin W. L. Keogh, Jan Gajewski

**Affiliations:** ^1^Department of Biomechanics, Wroclaw University of Health and Sport Sciences, Poland; ^2^Sport and Exercise Science Research Centre, School of Applied Sciences, London South Bank University, UK; ^3^Faculty of Health Sciences and Medicine, Bond University, Gold Coast, Australia; ^4^Sports Performance Research Centre New Zealand, AUT University, Auckland, New Zealand; ^5^Cluster for Health Improvement, Faculty of Science, Health, Education and Engineering, University of the Sunshine Coast, Australia; ^6^Kasturba Medical College, Mangalore, Manipal Academy of Higher Education, Manipal, Karnataka, India; ^7^Human Biology, Józef Piłsudski University of Physical Education, Warsaw, Poland

## Abstract

Stiffness, the resistance to deformation due to force, has been used to model the way in which the lower body responds to landing during cyclic motions such as running and jumping. Vertical, leg, and joint stiffness provide a useful model for investigating the store and release of potential elastic energy via the musculotendinous unit in the stretch-shortening cycle and may provide insight into sport performance. This review is aimed at assessing the effect of vertical, leg, and joint stiffness on running performance as such an investigation may provide greater insight into performance during this common form of locomotion. PubMed and SPORTDiscus databases were searched resulting in 92 publications on vertical, leg, and joint stiffness and running performance. Vertical stiffness increases with running velocity and stride frequency. Higher vertical stiffness differentiated elite runners from lower-performing athletes and was also associated with a lower oxygen cost. In contrast, leg stiffness remains relatively constant with increasing velocity and is not strongly related to the aerobic demand and fatigue. Hip and knee joint stiffness are reported to increase with velocity, and a lower ankle and higher knee joint stiffness are linked to a lower oxygen cost of running; however, no relationship with performance has yet been investigated. Theoretically, there is a desired “leg-spring” stiffness value at which potential elastic energy return is maximised and this is specific to the individual. It appears that higher “leg-spring” stiffness is desirable for running performance; however, more research is needed to investigate the relationship of all three lower limb joint springs as the hip joint is often neglected. There is still no clear answer how training could affect mechanical stiffness during running. Studies including muscle activation and separate analyses of local tissues (tendons) are needed to investigate mechanical stiffness as a global variable associated with sports performance.

## 1. Introduction

Stiffness is a quantitative measure of the elastic properties of the body and determines the ability to accumulate potential elastic energy. The concept of stiffness was developed in classical mechanics to describe the behaviour of elastic deformable bodies under application of external forces. In the seventeenth century, the British physicist Robert Hook stated a proportional relationship between the magnitude of the deforming force (*F*) and the deformation (Δ*l*) of the body. Therefore, as a part of Hooke's law, stiffness (*K*) was defined as a ratio of the amount of deforming force (or force change) to the unit of deformation (or as a ratio of the amount of deforming torque to the angle of deformation for rotational motions) [1–3].

Elastic deformable bodies have the ability to recover the previous shape and volume (i.e., they return to their initial size) after mechanical forces that cause deformation are removed. These deformations are fully reversible. Due to the influence of external deforming forces, the elastic bodies accumulate potential elastic energy, which they release back to the system when returning to the original length. The work performed by the deforming forces equals the value of the potential elastic energy accumulated in the spring compliance elements (assuming there are no energy losses due to friction and resistance forces) [2, 3].

The ability to absorb and return potential elastic energy is also observed in the musculotendinous groups in the human body. The potential elastic energy stored by the passive structures (tendon and aponeurosis) during contractile cycle of a muscle, e.g., during lengthening of the entire muscle-tendon unit, can increase the energy supplied by the compliant tissues during the proceeding shortening phase. Consequently, the substantial capacity of the tendon and aponeurosis to store elastic strain energy can enhance the total mechanical energy produced by the muscle-tendon unit during the concentric phase of muscle work or reduce muscle fibre work and metabolic energy expenditure. Potential elastic energy stored in muscle-tendon units reduces the metabolic energy spent by muscles responsible for movement in specific joints and is associated with the change in the kinetic energy of the body being moved [3–7]. Therefore, stiffness, the quantitative measure of the resistance offered by an elastic body to deformation, may be an essential factor in the optimization of human locomotion, because it is related to the maximal performance of cyclic and single dynamic movements [1, 8, 9].

However, the strict concept of stiffness has been introduced for relatively simple passive bodies (they maintain constant shape if external deforming forces are absent or sustainable). A human muscle (as a whole) does not behave like a passive body with linear force-deformation characteristics [2]. The muscle-tendon complex consists of two elements of different stiffness connected in series. A muscle is made of force-producing active (contractile) components and passive components (serial and parallel elastic elements) consisting of tendons, fascia, and other connective tissues, each with different biomechanical properties [10]. The magnitude of the forces (and mechanical power) generated depends on muscle activation, muscle length and its velocity, and on the use of elastic elements, which increase the effectiveness (and efficiency) of contractile elements. Tendon stiffness increases with lengthening [11] (due to the toe region in tendons' force-length relationship), and muscle stiffness increases with muscle lengthening or tension (activation level) [12]. However, while tendon stiffness is relatively constant, muscle stiffness is greatly influenced by the force developed [12]. The stiffness of a muscle increases the more motor units of the muscle which are activated [13]. Thus, the stiffness of the entire muscle-tendon complex varies and depends to the greatest extent on the stiffness of the muscle. It can be concluded that the activity of the muscles allows the potential elastic energy to be stored in the tendons since at the same deformation of the entire spring complex, the greater part of energy goes to less stiff element. Muscle tension is a factor regulating the stiffness of the support limb during locomotion and jumps. The coactivation of extensors and flexors in the moment preceding contact with the ground is aimed at regulating the “leg-spring” stiffness and preparing the limb to transfer the anticipated forces in the contact phase [14]. Muscle stiffness increases in eccentric phase, when the stretch reflex generates an extra activation. A musculotendinous unit is capable of resisting higher passive tensile forces when it is in a lengthened position or when it is stretched. In an active muscle state, the shape of generated muscle force over the entire physiological range of movement is not the same for every muscle as muscles in vivo can operate at different regions of the force-length relationship [15–17]. Moreover, body parts may change configuration in relation to each other (displacement) and not be deformed at all (like a passive bodies). Change in muscle length (deformation) can be caused by the action of contractile elements or external forces. Therefore, length of an active muscle or joint angle can change without a contribution of deforming forces. Consequently, it is possible to obtain the same magnitude of force at different joint angles and different force values at a specific joint angle [2]. Therefore, using the concept of stiffness in locomotion and performance analyses for much more complex biological objects than simple passive bodies is associated with numerous conceptual difficulties.

Stiffness should be understood as the resistance does not depend on time, velocity, or acceleration, but only on the displacement (for a passive elastic body with linear force-deformation characteristics, the value of stiffness will be the same at a relatively low or high level of deformation). The proper measurements of stiffness are performed during steady-state body deformation (from one equilibrium state to another equilibrium state). If stiffness measurements are not performed during steady-state body deformation but during transient states, the substantial value of *dF*/*dl* might contain components originating from inertial forces and damping. Therefore, the variable measured in the above case is not stiffness viewed in strict mechanical terms due to the substantial contribution of other factors that affect the *F*(Δ*l*) relationship, especially during transient states. In locomotion analyses when the body is in motion, certain “varieties” of stiffness are used [2, 3].

With respect to living bodies, the mechanical stiffness can be divided into quasi-stiffness and joint stiffness. Latash and Zatsiorsky [18] defined quasi-stiffness as the ability of the human body to oppose external displacements with disregard to displacement profile over time. Leg and vertical stiffness are the most frequently used types of quasi-stiffness in human and animal locomotion analysis to describe the mechanical properties of a “spring” representing the lower limbs (according to the assumptions of body modelling as a spring-mass model, which contains a massless supporting “leg-spring”, a material point representing the total body mass, and a parallel source of force resulting from the active action of the muscles involved in the take-off) [1, 19]. Leg quasi-stiffness is understood as the ratio of changes in the ground reaction force to the respective changes in “spring length” representing both lower limbs, whereas vertical quasi-stiffness is understood as the ratio of changes in the ground reaction force to the respective vertical displacement of the centre of mass (COM). Unfortunately, these two distinct stiffness concepts are often confused and consequently used interchangeably or incorrectly [20]. Joint stiffness is resistance to displacement within a given joint (e.g., hip, knee, or ankle) and depends on the mechanical properties of the movements related to this joint and all structures involved in this movement [2, 9, 21]. Research analysing leg, vertical, and/or joint stiffness have typically been conducted during cyclic (e.g., walking, running, or hopping) and single (e.g., vertical jumps) locomotor movements.

The relationships between mechanical stiffness (leg, vertical, and joint) and movement performance are areas of interest to the sport and research communities. Several authors have already tried to organise an understanding of stiffness in their review articles [1, 6, 9, 18, 21–30]. However, the multiple definitions and equations used to define vertical, leg, and joint stiffness along with advances in research into the topic leave the relationship between stiffness and movement performance are still not fully explored. The practice of sports training reveals some questions regarding the role of potential elastic energy and stiffness as a key factor responsible for determining performance. The reason for this may be the lack of longitudinal studies that have investigated the effects of strength or power training on mechanical stiffness and consequently the relative lack of concrete recommendations that would allow to improve the speed-strength abilities of an athlete and their competitive sport results. The speculations concerning a desirable value of “leg-spring” stiffness that is the most advantageous for the accumulation of potential elastic energy and most favours reaching maximal sport performance have been partially examined [1, 3, 22, 24–28, 31–35]. However, no studies have provided unequivocal evidence for the presence of a desired value of “leg-spring” stiffness. Moreover, the conceptual and methodological confusion surrounding stiffness makes it difficult to organise the knowledge and compare the results obtained in the past research.

Some reports refer to changes in stiffness under the influence of sports training (e.g., plyometric or isometric). However, they take into account the stiffness of local structures (e.g., tendon) [36–46]; the determination of which may be more complicated than the discussed values of leg, vertical, and joint stiffness. Several reports analysed the relationships between mechanical (leg, vertical, or joint) stiffness and movement performance (e.g., during biomechanical types of jumps) before and after the applied training program. However, they did not concern the sport-specific movements, such as running [42, 47–50]. Chelly and Denis [51] reported on positive relationships between maximal running velocity during 40 m sprint and vertical stiffness during hopping task. Bret et al. [52] found that athletes with greater vertical stiffness obtained higher acceleration between the first (0–30 m) and the second (30–60 m) intervals during 100 m sprint performance and presented a larger deceleration between the second and the third intervals (60–100 m). However, vertical stiffness was also determined based on the hopping test. It seems that these findings would be much more valuable if the stiffness was also measured during running. Lorimer et al. [53] reported that comparability of stiffness (leg, vertical, and joint) during hopping and running was at most moderate.

It would be expected that a stiffer “leg-spring” may increase athletic performance by enhanced utilisation of potential elastic energy. Therefore, the aim of this overview is to examine the relationships between mechanical stiffness (leg, vertical, and joint) and running performance, both in cross-sectional and training studies. Such a review is important as many studies assessing stiffness in humans have focused on jumping or hopping motions that are not commonly performed in sporting events, with the majority of the studies being cross-sectional in design. This review may provide additional insight regarding how different stiffness values obtained from running tasks may be representative of common sporting locomotor activities and how training-related changes in stiffness characteristics may underpin improvements in running performance.

## 2. Materials and Methods

A search of the PubMed and SPORTDiscus (EBSCO) bibliographic electronic databases was conducted in October 2020. The search terms used included (“leg” OR “lower limb” OR “lower extremity” OR “vertical” OR “joint”) AND (“stiffness”) AND (“run∗” OR “sprint∗” OR “jog∗”) AND (“sport”). Review and original empirical research articles and other related literature were selected based on the title and abstract. Additionally, Google Scholar, ResearchGate, and the reference lists of articles found were also checked to ensure no relevant studies were omitted during searching process. The following criteria were considered:

- Papers written in English only
- Studies with human samples
- No duplicates (papers found from several sources)
- No publication time restriction

Only studies which had measures of mechanical (leg, vertical, or joint) stiffness during running performance were included in further analysis. Studies describing other human movements (e.g., hopping), studies analysing the type of footwear, studies which failed to determine stiffness during the running performance (e.g., using oscillation technique, ultrasonography, or dynamometers or during other types of movement), and modelling-based studies or those concerning different types of stiffness than mechanical have been omitted. After a detailed review of the full texts, 92 meet all the criteria (Figure 1) with a publication date between 1980 and 2021 (the range of the year's results from the selection process conducted). There were a number of papers that measured more than one type of stiffness and were therefore discussed in several subsections. The number of papers described mechanical stiffness was 68 for leg stiffness, 65 for vertical stiffness and 23 for joint stiffness.

## 3. Results and Discussion

### 3.1. Quasi-Stiffness during Running Tasks

Running is a complex motion that engages the whole body and it occurs in various forms in track and field competitions or team sports games. Depending on the running distance, it is necessary to either reach submaximal velocity and cover the distance in the shortest possible time or keep the desired velocity for a certain distance. The running distance is covered through cyclic lower limb movements based on continuous acceleration and deceleration phases. Therefore, human running performance is similar to the motion of a bouncing ball (the so-called “bouncing gait”) and can be considered in accordance with the assumptions of spring-mass model (in which the lower limbs perform the role of “springs” responsible for the COM movement). Leg and vertical stiffness are commonly used to describe the mechanical properties of a “leg-spring” representing the lower limbs during running task [3].  Figure 2 shows a simple spring-mass model that can be used to determine quasi-stiffness (leg or vertical) during vertical displacements only. The modification of the spring-mass model presented in Figure 3 also includes horizontal displacements. Therefore, leg and vertical stiffness can be estimated for vertical and horizontal movements. However, vertical stiffness only considers vertical body displacements. Leg stiffness (*K*_leg_) and vertical stiffness (*K*_vert_) are expressed by the following equations:

(1) $$\begin{array}{c} K_{\text{leg}}=\frac{F}{\Delta L},\\ K_{\text{vert}}=\frac{F}{\Delta y}, \end{array}$$

where *F* is the deforming force (the causes of the change in deformation), Δ*L* denotes the change in “leg-spring” length (deformation), and Δ*y* is the displacement of COM (deformation). However, if the relationship between the deforming force and the deformation is nonlinear or deformation is plastic, the derivative (*d*) from Equations (2) or (3) should be used [2]:

(2) $$\begin{array}{c} K_{\text{leg}}=\frac{dF}{dL}, \end{array}$$

(3) $$\begin{array}{c} K_{\text{vert}}=\frac{dF}{dy}. \end{array}$$

The work performed by the deforming forces *F* equals the value of the potential elastic energy accumulated in the spring compliance elements. Potential elastic energy is proportional to the square of deformation and can be given by the following equation:

(4) $$\begin{array}{c} E_{\text{pe}}=\frac{1}{2}∙K∙{\Delta l}^{2}, \end{array}$$

where *E*_pe_ is the potential elastic energy, *K* denotes the stiffness (longitudinal), and Δ*l* is the deformation (change in length, displacement).

If stride frequency is relatively constant or the acceleration of the runners COM is relatively low (relatively constant movement velocity), then quasi-stiffness (leg and vertical) does not significantly change during running [55–57]. Therefore, one of the most well researched topics to improve understanding of how quasi-stiffness is controlled during running is alterations in quasi-stiffness and other running variables with running velocity changes. Paradisis et al. [58] stated that quasi-stiffness (leg and vertical) are key to generating a higher top running velocity during a short sprint. Tables 1 and 2 list the studies on vertical and leg stiffness that meet the inclusion criteria.

#### 3.1.1. Vertical Stiffness

Vertical stiffness increases with running velocity and stride frequency [33, 55, 58–68] and body mass [69]. Vertical stiffness also increases with the level of maturity [70, 71]. However, Meyers et al. [72] reported a decrease in vertical stiffness with the level of maturity during 35 m sprint task. Arampatzis et al. [62] reported vertical stiffness values between 30.8 ± 8.1 and 93.0 ± 29.7 kN/m at running velocities from 2.6 ± 0.2 to 6.6 ± 0.2 m/s. Paradisis et al. [58] obtained vertical stiffness values between 73.8 ± 9.7 and 105.1 ± 16.8 kN/m at running velocities from 7.7 ± 0.3 to 9.4 ± 0.4 m/s, whereas Kuitunen et al. [59] noted values between 103 and 171 kN/m at running velocities from 6.7 to 10.3 m/s. Therefore, higher values of vertical stiffness would be expected to be reached during maximal sprinting than during slower running conditions. Paradisis et al. [58] reported that faster sprinters are characterised by shorter ground contact time, longer stride length, higher stride frequency, and greater vertical stiffness than slower sprinters during a 35 m sprint task. García-Pinillos et al. [66] also reported that elite level runners are characterised by greater vertical stiffness than novice runners during treadmill running at velocities from 6.2 to 11.2 m/s. Rumpf et al. [73] noted positive relationships between relative vertical stiffness and sprint velocity, vertical COM displacement, relative vertical peak force, and maximal “leg-spring” displacement during 30 m treadmill sprint.

An important factor that affects vertical stiffness and stride frequency is fatigue. Dalleau et al. [74] reported negative relationships between vertical stiffness and energy cost of running, as determined from the O_2_ consumption. Heise and Martin [75] concluded from the negative relationships between vertical stiffness and aerobic demand that less economical runners possess a more compliant “leg-spring” running style during ground contact phase. These findings may support the role of the mechanical stiffness in the metabolic energy cost of running at a given velocity (velocities: 3.35 m/s has been applied by Heise and Martin [75] and 5 m/s has been applied by Dalleau et al. [74]). Dutto and Smith [76] observed that runners decreased vertical stiffness and stride frequency during a moderate-intensity treadmill run to exhaustion. Changes in vertical stiffness were primarily associated with increases in vertical COM displacement, and not to changes in the peak vertical ground reaction force. The runners altered their running kinematics to allow for longer stride lengths and decreased stride frequency to maintain a constant running velocity. Decreases in vertical stiffness were proportional to decreases in stride frequency [76]. Hobara et al. [64] noted that vertical stiffness peaked at the 50-100 m interval and consistently decreased from the middle to the later part of the 400 m sprint. Morin et al. [55] reported that the decrease in 100 m sprint performance (decreased maximal and mean velocity) in fatigue conditions induced by the four repetitions of this running task was also accompanied by decreases in vertical stiffness and step frequency and increased ground contact time [55]. Girard et al. [56] showed that a decrease in running velocity in the last 50 m distance interval of a 100, 200, and 400 m sprint performances was accompanied by a decrease in stride length, stride frequency, and vertical stiffness and by an increase in ground contact time. The magnitude of decrement in vertical stiffness increased with sprint distance [56]. Other studies have also discovered significant relationship between decrements in both stride frequency and vertical stiffness and a progressive slowing in running velocity after two sets of five 5 s sprints [77], three sets of five 5 s sprints [57], six 20 m sprints [78], twelve 40 m sprints [79], six 30 s runs at 5.5 m/s [80], and during running anaerobic sprint test (RAST test, 6 × 35 m) [81]. Therefore, it can be concluded that fatigue causes decreased vertical stiffness during running tasks, resulting in lower efficiencies of movement with a concomitant increase in metabolic cost. Athletes characterised by enough high vertical stiffness during running may execute running tasks more economically (with less vertical COM displacements) and with higher performance through gaining a greater potential elastic energy return from musculotendinous structures.

It is also possible to change (decrease) leg and vertical stiffness by running with different (increased) knee flexion (the so-called “Groucho running”). This type of running technique lowers ground reaction forces and reduces flight time, but requires increased metabolic power (oxygen consumption) [82–85]. The above phenomenon should be taken into account in particular by team sport games coaches, where technique like “Groucho running” is often used. This running style is necessary to minimise flight time and therefore to maximise the potential to decelerate and change direction quickly.

#### 3.1.2. Leg Stiffness

In contrast to vertical stiffness, leg stiffness (with increasing running velocity) remains relatively constant or changes (increase) to a smaller extent during running [33, 55, 56, 58, 61–63, 65–68, 81]. However, leg stiffness increases with the level of maturity [70, 71]. Arampatzis et al. [62] reported leg stiffness values between 25.3 ± 4.2 and 35.2 ± 4.3 kN/m at running velocities from 2.6 ± 0.2 to 6.6 ± 0.2 m/s. Paradisis et al. [58] obtained leg stiffness values between 12.7 ± 2.3 and 15.5 ± 2.7 kN/m at running velocities from 7.7 ± 0.3 to 9.4 ± 0.4 m/s. Paradisis et al. [58] reported that faster sprinters are characterised by greater leg stiffness than slower sprinters during 35 m sprint task. In contrast, García-Pinillos et al. [66] observed that leg stiffness has similar values in elite and novice runners during treadmill running at velocities from 6.2 to 11.2 m/s. Rogers et al. [86] reported that leg stiffness has relationships with running economy (negative) and maximal sprinting velocity (positive).

However, it is possible to change leg stiffness value more than twofold by increasing stride frequency at a given running velocity [33]. Therefore, humans can change the stiffness of the “leg-spring” during running tasks, which can be useful, for example, when running on a variety of surfaces with different stiffness. Runners can adjust leg stiffness for their first step on a surface with different compliances allowing them to maintain similar running mechanics on different surfaces [87, 88]. By comparison with a hard surface, if the surface is soft and compliant, more time is required to reverse the COM downward velocity and perform take-off [89]. Stafilidis and Arampatzis [90] observed that surfaces of different compliances (stiffness from 550 to 5500 kN/m) did not have any clear effect on 60 m sprint performance and on the leg and vertical stiffness values. However, as the optimal track stiffness may be influenced by each of the runners' inherent stiffness characteristics, their shoes, and key running spatiotemporal characteristics, the lack of any clear association between track stiffness to running performance is not necessarily unsurprising [90].

In contrast to vertical stiffness, leg stiffness is not strongly related to the aerobic demand of running and fatigue [55–57, 76, 80, 81, 91–98]. The exceptions are the run to exhaustion at the velocity at VO_2max_ [99–102] and 60 min time trial run [103] during which leg stiffness decreases and vertical stiffness remains relatively constant. Dutto and Smith [76] reported that leg stiffness decreased initially from the beginning to 25% duration time in moderate-intensity treadmill run to exhaustion and then remained relatively constant. Decrease in leg stiffness was associated with increased changes in “leg-spring” length during ground contact phase and with decrease in the peak vertical ground reaction force [76]. Li et al. [104] reported a negative relationship between running economy and leg stiffness. Hobara et al. [64] noted that leg stiffness peaked at first 50 m interval and remained constant from next 50 m interval to finish during 400 m sprint. Morin et al. [55] found that leg stiffness and peak vertical ground reaction force remained relatively constant in fatigue conditions induced by four repetitions of 100 m sprints. Similar conclusions were obtained by Brocherie et al. [81] during RAST test with additional accompanying decrease in stride frequency and increase in ground contact time. Leg stiffness decreases during the last 50 m distance interval of a 100, 200, and 400 m sprint performances which were smaller than decreases in vertical stiffness and limited to 200 and 400 m tasks [56]. Other studies confirm that decreases in leg stiffness due to fatigue-induced reduction in sprinting velocity were much smaller than decreases in vertical stiffness [55, 57, 78, 79, 105–107].

At relatively low running velocity, runners predominantly hit the ground with the heel (heel strike), whereas at higher running velocity (sprinting), the foot strike is usually performed with the forefoot [59, 108]. Rearfoot strike pattern runners touching the ground with heel and using a rolling foot strategy result in increased ground contact time. In contrast, forefoot runners immediately shift from energy absorption phase to the propulsion phase which will decrease ground contact times and hence increase the rate of the ground reaction force application [109]. Therefore, using the forefoot strike pattern may also be more beneficial to team sport players than rearfoot strike pattern. Forefoot strike pattern runners are characterised by greater leg stiffness, greater peak vertical ground reaction force, shorter contact time, and smaller “leg-spring” change compared with rearfoot strike pattern runners [109].

Leg stiffness is also likely to influence the ability to effectively execute change of direction tasks. Greater leg stiffness allows to less loss of velocity when changing direction [110]. An inability to preplan a side-step cutting manoeuvre may result in a greater decrease in velocity and reduce cut angle. Reduced preplanning time available for side-step cutting increased leg stiffness. Moreover, unanticipated cutting significantly increased leg stiffness compared to the anticipated cutting [110].

The difference in behaviour between vertical stiffness and leg stiffness during running tasks is potentially due to the fact that leg stiffness is mainly determined through the mechanical properties and activation of lower limb musculotendinous system with only small “leg-spring” stiffness variations depending on velocity. Vertical stiffness is not only reliant on the properties and activation of the lower limb but also on the whole body [22]. Moreover, COM displacement depends on the spatial position of each body part, including the upper limbs. The total mass of the body (COM) is not concentrated at the upper end of the “leg-spring”. Therefore, the displacement of the COM is not the same as the displacement of the upper end of the “leg-spring” [3]. Differences between leg and vertical stiffness may also be due to the hip joint displacement. It has a much smaller effect on vertical stiffness.

### 3.2. Joint Stiffness during Running Tasks

Quasi-stiffness is a concept that considers the limb (leg stiffness) or body (vertical stiffness) as a whole system rather than only the musculotendinous system. Therefore, quasi-stiffness also depends on the stiffness of other tissues, such as ligaments, blood vessels, and bones. The elastic properties and the ability to accumulate potential elastic energy are different for each of these tissues [2]. However, the “leg-spring” model is dependent also on hip, knee, and ankle kinematics. Therefore, the torsional spring model offers a different view of “leg-spring” stiffness than the spring-mass models. By using the torsional spring model, it is possible to estimate the joint stiffness values of the main joints of lower limb during vertical and horizontal movements.  Figure 4 shows an example of the torsional spring model that can be used in the determination of ankle, knee, and hip joint stiffness during vertical and horizontal displacements.

For rotational motions, joint stiffness (*K*_joint_) is expressed by the following equation:

(5) $$\begin{array}{c} K_{\text{joint}}=\frac{M}{\Delta \alpha }, \end{array}$$

where *M* denotes the deforming torque and Δ*α* is the angle of deformation. However, if the relationship between the deforming torque and the angle of deformation is nonlinear or deformation is plastic, the derivative (*d*) from Equation (6) should be used [2]:

(6) $$\begin{array}{c} K_{\text{joint}}=\frac{dM}{d\alpha }. \end{array}$$

The analysis of lower limb joint springs (hip, knee, and ankle) offers a different view of “leg-spring” stiffness than the quasi-stiffness.  Table 3 lists the studies on joint stiffness that meet the inclusion criteria. Unfortunately, only a few manuscripts consider all three lower limb joint springs or even hip joint stiffness [53, 112–114]. Hip joint stiffness increases with running velocity [113]. Jin and Hahn [113] stated that hip joint has a crucial role during swing phase for work and power generation.

#### 3.2.1. Knee and Ankle Joint Springs

Knee joint stiffness increased with running velocity [59, 62, 113, 115, 116]. Arampatzis et al. [62] reported knee joint stiffness values between 6.8 ± 4.1 and 19.1 ± 8.9 Nm/° at running velocities from 2.6 ± 0.2 to 6.6 ± 0.2 m/s. Kuitunen et al. [59] obtained knee joint stiffness values between 17 and 24 Nm/° at running velocities from 6.7 to 10.3 m/s. Knee joint stiffness during initial ground contact increases also with running velocity [116]. Tam et al. [115] reported that knee joint stiffness has positive relationships with rectus femoris activation and rectus femoris : biceps femoris coactivation ratio. Jin and Hahn [113] stated that knee joint has a crucial role during swing phase for energy absorption.

In turn, ankle joint stiffness (with increasing running velocity) remains relatively constant or changes (increase) to a smaller extent compared to knee joint stiffness [59, 62, 115, 117, 118]. Stefanyshyn and Nigg [117] and Kuitunen et al. [59] argued that ankle joint stiffness is dependent on the task activity rather than on the individual. Arampatzis et al. [62] reported ankle joint stiffness values between 16.4 ± 5.5 and 20.5 ± 8.2 Nm/° at running velocities from 2.6 ± 0.2 to 6.6 ± 0.2 m/s. Stefanyshyn and Nigg [117] reported ankle joint stiffness values of 5.7 Nm/° in running at 4 m/s and 7.4 Nm/° in sprinting at velocities from 7.1 to 8.4 m/s. Aeles et al. [119] did not obtain significant differences in ankle joint stiffness between young and adult well-trained sprinters during 10 m sprint (first stance phase). Charalambous et al. [120] noted a positive relationship between ankle joint stiffness on the ascending limb and the horizontal COM velocity at the end of the first stance phase. Kuitunen et al. [59] reported a negative relationship between ankle joint stiffness and ground contact time. Jin and Hahn [113] stated that ankle joint has a crucial role during stance phase for energy generation in running. Higher ankle joint stiffness results in more positive work performed and power generation [113].

Larger peak moment and mechanical power values at the ankle and knee joints are observed with increasing running velocity [62]. Running velocity also influences the change in the angle at the ankle and knee joint [62]. With increasing running velocity, larger changes are observed in the knee joint stiffness than in the ankle joint stiffness [59, 62]. Therefore, the increase in “leg-spring” stiffness may be mainly caused by the increase in knee joint stiffness. Joseph et al. [121] stated that knee joint mechanics may be altered to maintain consistent levels of leg and vertical stiffness. Arampatzis et al. [62] suggested that with increasing running velocity, the athletes alter the knee joint stiffness first. In accordance with the assumptions of the torsional spring model, “leg-spring” stiffness depends on the stiffness of three joint springs (in the ankle, knee, and hip joint). The contribution to the overall “leg-spring” stiffness of each joint spring is different. According to Equation (7), the greatest contribution to the overall stiffness value of the “leg-spring” will have the most compliant joint spring:

(7) $$\begin{array}{c} K_{\text{leg}‐\text{spring}}=\frac{1}{\left(1/K_{\text{ankle}}\right)+\left(1/K_{\text{knee}}\right)+\left(1/K_{\text{hip}}\right)}, \end{array}$$

where *K*_leg−spring_ is the “leg-spring” stiffness, *K*_ankle_ denotes the ankle joint stiffness, *K*_knee_ is the knee joint stiffness, and *K*_hip_ is hip joint stiffness.

Therefore, depending on the running velocity, theoretically, knee joint stiffness or ankle joint stiffness will have the most influence of overall “leg-spring” stiffness. Ankle joint spring should be more compliant than knee joint spring during substantial running velocity (sprinting). Günther and Blickhan [122] concluded that the knee joint is always stiffer and more extended than the ankle joint. However, this statement only seems true from a certain running velocity and may depend on the running technique [62].

Lower ankle joint stiffness and greater knee joint stiffness were associated with lower oxygen consumption during constant velocity running. More economical runners are characterised also with short ground contact times and greater stride frequencies [123]. Weir et al. [98] reported that knee joint stiffness increased and ankle joint stiffness decreased with running time during a prolonged treadmill run. Moreover, Melcher et al. [124] noted that oxygen consumption, ankle joint moment, and knee joint stiffness were greater during imposed forefoot strike pattern compared with rearfoot strike pattern. Therefore, the foot strike angle can also influence joint stiffness [124–126]. Change in foot strike pattern from rearfoot strike to midfoot strike may cause a decrease in ankle joint stiffness and increase in knee joint stiffness [126]. Melcher et al. [124] noted that knee joint range of motion, knee joint moment, and ankle joint stiffness were lower during imposed forefoot strike compared with rearfoot strike pattern.

### 3.3. The Effect of Training on Mechanical Stiffness

The assessment of training effects in runners seems to be the most correct when it is carried out with the use of running tests. Therefore, the possible changes in mechanical stiffness can then be determined based on a measurement during running.  Table 4 lists the longitudinal studies that meet this criterion. Nagahara and Zushi [127] have examined well-trained male athletes during 60 m sprints before and after a 6-month winter training session (combining of plyometric, sprint, weight, circuit, and individualised trainings). However, the participants specialized in different events (including a sprinter, two jumpers, five pole vault jumpers, and a decathlete) and followed their own training plans during the winter training period. Nagahara and Zushi [127] reported that the development of maximal velocity sprinting performance through longer step length was accompanied by increases in vertical and ankle joint stiffness, although leg and knee joint stiffness remained constant. Ache-Dias et al. [128] reported that the addition of 4 weeks of jump interval training into a continuous endurance treadmill training program induced an increase in the stiffness (leg and vertical) and stride frequency and a decrease in stride length. However, these changes do not affect running economy. Lum et al. [129] noted that 6 weeks of intermittent sprint training and plyometric training led to improvement in 10 km performance in moderately trained endurance runners despite reduction in weekly training mileage. The improvement in running performance was accompanied by an increase in power, whereas leg and vertical stiffness remained relatively constant. Similarly, Roschel et al. [130] did not report changes in vertical stiffness in recreational runners after 6 weeks of resistance training or whole-body vibration training.

In contrast, Rumpf et al. [73] observed decreases in 30 m treadmill sprint time, relative leg stiffness, and relative vertical stiffness in youth after 6 weeks of resisted sled towing training. Stride frequency, average power, peak horizontal force, average relative vertical forces, and vertical displacement increased. While this study reported decreased sprint times, the decrease in stiffness might be viewed as disadvantageous in the long term as these reductions in stiffness may actually increase foot contact time and result in a reduction in stride frequency and ultimately running speed.

While McMahon et al. [26] and Brazier et al. [22] have recommended that in terms of training to increase “leg-spring” stiffness, resistance training should be performed with loads above 75% of 1 repetition maximum and should precede high-intensity plyometric and power training, there is still no clear answer how training could affect mechanical stiffness during running due to a very small number of studies on this topic. Papers that did not assess mechanical stiffness changes (caused by training) during running task were omitted from this review. Perhaps due to the increase in rate of force development, some power (plyometric) training would result in an increase in mechanical stiffness. However, it is not known how power training affects leg, vertical, or joint stiffness during running, although it is presumably known how mechanical stiffness changes might affect running performance. Moreover, there is a lack of studies on training effects in elite athletes. There is also the question of obtaining the possible desired “leg-spring” stiffness value under the influence of training.

### 3.4. Desired “Leg-Spring” Stiffness

The total mechanical energy involved in human body movement is the sum of kinetic and potential energy. With each running stride, the kinetic energy change of horizontal motion (related to the braking action of the ground) and the gravitational potential energy change due to the (vertical) displacements of the runners COM. Potential elastic energy is associated with the change in the kinetic energy of the body being moved. Due to braking and lowering of the runners COM in the initial part (absorption) of the ground contact phase during running, the decrease in the kinetic energy and gravitational potential energy is partially stored in the form of potential elastic energy by the stretched musculotendinous groups. The ability of the musculotendinous groups to store and return potential elastic energy increases the mechanical energy supplied by active contracting muscles used in the take-off phase. Consequently, the total mechanical energy supplied by the entire muscle-tendon unit during the propulsion phase can obtain greater values and/or less work needs to be performed by the muscles' contractile elements [3, 6]. A certain amount of “leg-spring” stiffness is required for effective storage and utilization of potential elastic energy in the musculotendinous groups during “stretch-shortening cycle” (SSC) movements, such as running [22]. Greater stiffness of the “leg-spring” provides the capacity to store more potential elastic energy during the ground contact phase. Therefore, it would be expected that higher (or high enough) values of mechanical stiffness (leg, vertical, and joint) may also increase running performance and/or execute running tasks with more mechanical economy. Cavagna et al. [131] suggested that the role of potential elastic energy becomes more important in sprint tasks at running velocities greater than 7 m/s, although its contribution to lower velocity running is also of importance.

The total “leg-spring” involves many skeletal muscles and tendons and other passive structures. These tissues can be stretched and recoil and consequently accumulate potential elastic energy during these actions [32]. During running with relatively low velocity, ankle plantar flexors contribute the majority of the force necessary for vertical support and horizontal propulsion, whereas the quadriceps muscle group is the largest contributor to horizontal braking of the runners COM and vertical support during the early stage of the ground contact phase [132]. The gluteus maximus, quadriceps, and ankle plantar flexors are the major contributors to acceleration of the body COM during running [132, 133]. The muscles are activated before the lower limb hits the ground, therefore reducing the amount of muscle stretch during initial ground contact and absorption (braking) phase [32]. However, to generate sufficiently large ankle joint torques, the ankle plantar flexor muscles shorten throughout the entire ground contact phase (or work in quasi-isometric conditions during the early part of the ground contact phase), despite the entire musculotendinous units undergoing a SSC [134]. Most of the stretch can be taken up by the tendons, resulting in potential elastic energy storage in these spring elements [32]. The musculotendinous system design of the ankle plantar flexors supports the storage and utilization of tendon elastic strain energy over muscular work [134, 135]. In muscle-tendon units with long compliant tendons (such as the Achilles tendon), the tendons can store a high amount of potential elastic energy; therefore, during the push-off phase, less work needs to be performed by the muscles due the energy returned by the tendons. For example, the Achilles tendon, which is long and compliant, is able to contribute about 35% of the mechanical energy necessary for performing each running stride (obviously, the entire “leg-spring” is formed also by other soft tissues with elastic properties) [32]. The compliance of the serial elastic elements allows the muscle fibres to contract at preferred velocities for maximal power output and efficiency (according to force-length curve) and allows to deactivating fibres during shortening periods. Therefore, the muscle fascicles shorten at a much slower velocity (often very different from the velocity of the whole musculotendinous units) with high velocity shortening during take-off in running achieved by recoil of the serial elastic elements [134, 136, 137].

For a given human body modelled as a spring-mass system (with specific body mass, leg-spring length, the horizontal and vertical landing velocities, and leg-spring swept angle), some particular value of the “leg-spring” stiffness may hypothetically be the most beneficial for movement performance. Greater or lower “leg-spring” stiffness compared to desired values can cause the lower limbs to partially lose elastic capacity, which will have a negative effect on the accumulation and utilization of elastic energy. If the “leg-spring” is too stiff, the body may take-off too soon reducing the capacity to improve flight time through addition of muscular force. If the “leg-spring” is too compliant, the body may rise too late with considerable energy lost through relaxation of the elastic tissue, thereby reducing the advantage for the musculotendinous system during the SSC [20].

“Leg-spring” stiffness is expected to be greater in athletes than nonathletes during running tasks. With similar changes in the length of the “leg-spring”, athletes release greater force than nonathletes. Therefore, increases in “leg-spring” stiffness make it theoretically possible for runners to absorb greater loads, as a higher level of deforming force (torque) is required to perform joint movement. This phenomenon may be important in training, as it allows for working with higher loads. However, based on the analysis of vertical jumps, it seems that the desired “leg-spring” stiffness value is relatively small in relation to the “maximum” [3].

Greater accumulation of potential elastic energy may occur by increasing stiffness and/or deformation. However, according to Equation (4), increases in deformation seem more beneficial because the value of potential elastic energy depends on the squared length change. Therefore, theoretically smaller “leg-spring” stiffness allows “leg-spring” length change by using a lower force and consequently greater length change can be obtained, which should increase the accumulated potential elastic energy. However, the “leg-spring” length change cannot be too excessive (beyond the desired range of lower limb joint flexion during ground contact phase), as such changes would result in large increases in ground contact time and decreases in step frequency. After reaching an “optimal” lower limb joints flexion angle, further increases in the accumulated potential elastic energy are possible by increasing stiffness. “Leg-spring” stiffness will increase with increased deforming force at “optimal” lower limb joint flexion angles during running tasks [3].

Because athletes are able to generate a greater ground reaction force than nonathletes, their maximum “leg-spring” stiffness is greater. Therefore, a relatively low “leg-spring” stiffness will be greater for an athlete than for a nonathlete. The greater value of “leg-spring” stiffness in athletes (in comparison to nonathletes) will be (on the condition that the desired range of motion in the lower limb joints is obtained) an additional factor that increases the accumulated potential elastic energy and, consequently, performance. Therefore, the desired “leg-spring” stiffness value can be an individual variable property [3].

The speculations concerning a desirable value “leg-spring” stiffness that is the most advantageous for the accumulation of potential elastic energy and most favours reaching maximal sport performance have already been addressed in many previous studies [1, 3, 22, 24–28, 31–35]. However, no studies have provided unequivocal evidence for the presence of a desired “leg-spring” stiffness value. Because desired “leg-spring” stiffness can be influenced by task, and individual and environmental factors, the estimation of this desired value and determination of how this value might be influenced by changes in stiffness at each joint spring may prove to be extremely difficult.

### 3.5. Limitations and Other Important Factors

#### 3.5.1. Computation Methods

The studies included in this review utilised several computational methods to estimate mechanical stiffness, with such approaches not always necessarily yielding the same values [1, 21, 24, 53, 62, 122, 138–143]. Therefore, it may be important to be aware of these between-study differences, meaning that analysing the profile of the force-displacement (or torque-displacement) curve and the values of deforming force (torque) and displacement (change in length, deformation) may be useful. Estimation of the mechanical stiffness value does not always follow the force-displacement profile, and the displacement (of COM or “leg-spring” compression) during ground contact phase is defined in various ways. High magnitudes of deforming force and displacement at one hand and low magnitudes of deforming force and displacement on the other hand could both lead to similar stiffness values. Moreover, mechanical stiffness during running tasks has been evaluated during both treadmill and typical over ground effort conditions. It should be remembered that the measurements performed on the treadmill give slightly different values of kinematic and kinetic variables (including “leg-spring” stiffness) compared to the analysis carried out under field conditions [144].

Another important factor that seems necessary to take into account in stiffness estimation is body mass. A positive relationship between stiffness and body mass can result from maintaining the natural vibration frequency of the human body, which is dependent on internal elastic forces and inertia [7]. Therefore, the relationships of mechanical stiffness with the variables describing the running tasks may be different if the value of stiffness related to body mass is taken into account, not the absolute value [3, 65, 67, 145, 146].

Mechanical stiffness is commonly assessed in both laboratory and field tests. Regardless of the test mode, any stiffness test must be valid and reliable if the data can be used to inform training decisions. Pappas et al. [147] reported that leg and vertical stiffness, as well as related kinematic parameters, obtained using the sine wave method during treadmill running at 4.4 m/s, were highly reliable, both within and across days. However, Joseph et al. [148] reported that during 10 m overground running (at 3.8 m/s), vertical stiffness has good reliability, leg stiffness has moderate reliability, and knee and ankle stiffness has poor reliability. Leg stiffness [75] and knee joint stiffness [59] are characterised by substantial interindividual variations. Therefore, researchers may need to better demonstrate the validity and reliability of their stiffness measures, with consensus recommendations from experts warranted, perhaps similar to the SENIAM approach for electromyography data collection and analysis [149].

#### 3.5.2. Running Phases

There are several consecutive phases during running distance: start, push-off, acceleration, maximum velocity (or desired submaximal velocity for longer distances), and velocity maintenance [120]. All these running phases are characterised by different stride length-to-frequency ratios, technical and physiological demands that may require different “leg-spring” stiffness values to maximise performance and different training programs [120, 150–152]. This may indicate that different forms of training may be required to improve the stiffness characteristics relevant to each running phase.

Ground contact can be divided into absorption (braking) and propulsion phases, which differ in their characteristics and purpose [153]. This suggests that the mechanical stiffness during braking and propulsion phases does not necessarily have to be the same. To understand the phenomena occurring during running tasks, it seems necessary to determine the mechanical stiffness for both these phases separately [154, 155]. Such an approach has been used in a number of studies, although these approaches differ. Luhtanen and Komi [156] estimated vertical stiffness during running and long jump with a division into eccentric and concentric phases. Butler et al. [1] proposed to calculate joint stiffness with division into two separate phases: during the joint moment increase and during the joint moment decrease. Hunter [157] proposed separation of the heel strike part from the ground contact phase during running as a part with much greater stiffness compared to rest of ground contact phase. However, these approaches do not appear to be commonly used.

#### 3.5.3. Running Technique

The specific nature of each sport should also be considered in the analysis because running technique used by team sports players (like a “Groucho running”) differs significantly from track athlete technique [158]. It is important because running performance affects game performance indicators [159]. Team sport players (in soccer, rugby, football, basketball, handball, lacrosse, or field hockey) run with a relatively lower height of the COM, less knee flexion during swing phase, and lower knee lift. This technique helps team sport players to decelerate and change direction faster [158, 160]. The acceleration phase for team sport players is much shorter than that for track sprinters, and the maximal running velocity is reached earlier [161]. All of these factors may therefore alter the desired level of “leg-spring” stiffness for team sport players compared to track athletes. The type of footwear used by athletes and team sport players also may have some role in terms of altering the “leg-spring” stiffness and subsequent sporting performance [162–165]. The anatomical structure of the foot is another individual factor that can influence leg stiffness. High-arched runners have increased leg stiffness, knee joint stiffness, and ankle joint stiffness compared to low-arched runners [166–169].

## 4. Conclusions

Mechanical stiffness is a group of variables (leg, vertical, and joint stiffness) that seem to have an important role in running performance. Based on the reported positive relationships between mechanical stiffness and running velocity, a stiffer “leg-spring” should probably increase running performance and contribute to greater mechanical efficiency in running tasks. However, the positive relationship observed between mechanical stiffness and running velocity does not mean that the maximum possible “leg-spring” stiffness will be the most desirable. Therefore, while determining what is desired “leg-spring” stiffness value during running is perhaps the ultimate goal of such research; “optimal” stiffness values may differ somewhat based on differences in the individual, environment and exact running task performed in accordance with the constraints led approach to motor control [170]. This may explain why no studies have provided unequivocal evidence for the presence of a desired value of “leg-spring” stiffness for any particular running task or population group. As leg-spring stiffness values can be influenced by variations in the stiffness of all three lower limb joint springs (hip, knee, and ankle), the relative lack of analysis of all three lower limb joint springs significantly limits the current understanding of these joints' roles in modulating the mechanical stiffness behaviour during human running. There is still a very small number of studies that have examined training-related changes in mechanical stiffness, with only a small proportion of the studies examining the potential relationships to changes in running performance. Moreover, only a few works concern the analysis of spring-mass model properties performed on top-level athletes and players or over an entire running distance in field conditions with typical acceleration-deceleration running velocity pattern [55, 64, 93, 94, 171, 172].

The number of factors influencing mechanical stiffness during running makes it difficult to formulate clear and general conclusions about training recommendations. All three levels of constraint effecting the individual, environment, or task constraints including age, gender, running technique, sporting background, fatigue, running distance, and running surface should be taken into account. Until researchers investigate how mechanical stiffness can be altered with different forms of training, the influence of “leg-spring” stiffness on running performance will remain somewhat unclear. It seems that studies focusing on the analysis of local tissues (muscle, tendon) as well as more global phenomenon including the interaction of the central nervous and peripheral systems and how the plasticity of these systems affects their interplay with regard to “leg-spring” stiffness on running performance may allow for a better understanding of the running mechanics.

## Figures and Tables

**Figure 1:** Selection process of papers focused on mechanical stiffness during running [54].

**Figure 2:** An example of a simple spring-mass model used to estimate leg and vertical stiffness during vertical body displacements only, where COM denotes the centre of mass, Δ*L* is the change in “spring length” representing both lower limbs, Δ*y* is the displacement of COM, and GRF means the ground reaction force (based on Blickhan [19]).

**Figure 3:** An example of a spring-mass model used to estimate leg and vertical stiffness during running tasks, where COM denotes centre of mass, Δ*L* is change in “spring length” representing both lower limbs, and Δ*y* is displacement of COM (based on McMahon and Cheng [20]).

**Figure 4:** An example of torsional spring model used to estimate ankle, knee, and hip joint stiffness during running tasks, where *α*_ankle_ denotes the ankle joint angle, *α*_knee_ is the knee joint angle, and *α*_hip_ is the hip joint angle (based on Farley et al. [111]).

**Table 1:** List of the studies on leg stiffness during running.

Authors	Year	Number of participants	Sport background	Motor skill
Ache-Dias et al. [128]	2018	18 (males + females)	Recreational runners	Submaximal constant load running test on treadmill (6 min at 9 km/h)
Arampatzis et al. [62]	1999	13 runners	Not mentioned	Running at 2.5, 3.5, 4.5, 5.5, and 6.5 m/s
Avogadro et al. [138]	2004	13 runners	Healthy trained runners	3 min running on treadmill at 12, 14, 16, and 18 km/h
Bitchell et al. [97]	2019	7 + 13 runners	Trained + untrained runners	Incremental running on treadmill
Brocherie et al. [81]	2015	8 males	International football players	RAST test (6 × 35 m sprint)
Cavagna et al. [63]	2005	4 males + 1 female	Not mentioned	Running at different velocities (from 5.2 to 20.5 km/h)
Choukou et al. [106]	2012	8 males	Sprinters competing at the regional level	100 m sprint
Coleman et al. [141]	2012	19 males	Well-trained middle-distance runners	Running at different velocities (from 2.5 to 6.5 m/s)
Cronin and Rumpf [69]	2014	16 males	Young athletes	30 m sprint on treadmill
Dal Pupo et al. [107]	2017	21 males	Futsal players	10 m sprint
Dutto and Smith [76]	2002	11 males + 4 females	Well-trained runners	Running on treadmill to exhaustion at a velocity corresponding to 80% of the VO_2max_
Farley and González [33]	1996	4 males	Experienced treadmill runners	Running on treadmill at 2.5 m/s (while using a range of stride frequencies from 26% below to 36% above the preferred stride frequency)
Ferris et al. [88]	1999	6 females	Healthy	17 m running at 3.0 m/s
Ferris et al. [87]	1998	5 humans	Not mentioned	Running at 5 m/s
Fourchet et al. [102]	2015	11 males	Highly trained middle-distance runners	Running on treadmill to exhaustion at a velocity corresponding to 95% of the VO_2max_
García-Pinillos et al. [103]	2020	22 males	Endurance runners	60 min running on treadmill
García-Pinillos et al. [66]	2019	22 males	Novice and elite endurance runners	Incremental running on treadmill at 10, 12, 14, 16, and 18 km/h
Gill et al. [155]	2020	16 males + 12 females	Runners	32 m running at 3.3, 3.9, 4.8, and 5.6 m/s
Gindre et al. [83]	2016	77 males + 14 females	Healthy and active	50 m running at 3.3, 4.2, and 5.0 m/s
Giovanelli et al. [95]	2016	18 males	Ultraendurance runners	“Supermaratona dell'Etna”
Girard et al. [150]	2015	13 males	Team and racket sport background	3 × 5 s sprints on treadmill
Girard et al. [80]	2017	20 males	Field hockey players	6 × 30 s running on treadmill at 115% of the VO_2max_
Girard et al. [57]	2017	14 males	Recreationally intermittent sports	3 × 5 s sprints on treadmill + running on treadmill at 10 and 20 km/h
Girard et al. [56]	2016	11 males	Physical education students practicing a field sport	100, 200, and 400 m sprint on treadmill
Girard et al. [79]	2011	16 males	Recreational team or racket sports athletes	12 × 40 m sprints
Girard et al. [96]	2017	18 males	Physical education students	800 m running
Girard et al. [91]	2010	12 triathletes	Highly and well-trained triathletes	5000 m running at self-selected velocity
Girard et al. [93]	2013	12 males	National level triathletes	5000 m running at self-selected velocity
Girard et al. [78]	2011	13 males	Young soccer players	6 × 20 m sprints
Günther and Blickhan [122]	2002	8 males + 4 females	Sports students and active sportsmen	Running at convenience velocity (from 3.7 to 5.6 m/s)
He et al. [61]	1991	4 males	Healthy	Running on treadmill at 2.0, 3.0, 4.0, 5.0, and 6.0 m/s
Heise and Martin [75]	1998	16 males	Recreational runners	15 m running at 3.35 m/s
Hobara et al. [64]	2010	8 males	Well-trained sprinters and runners	400 m sprint
Hunter and Smith [105]	2007	11 males + 5 females	Recreational runners	1 h running on treadmill at constant velocity
Joseph et al. [148]	2013	20 males	Various sports	10 m running at 3.35 m/s
Joseph et al. [121]	2014	20 males	Various sports	10 m running at 3.35 m/s
Hayes and Caplan [101]	2014	6 runners	Subelite middle-distance runners	Running on treadmill to exhaustion at velocity corresponding to VO_2max_
Li et al. [104]	2021	28 males	Collegiate distance runners	Running at 12, 14, and 16 km/h
Liew et al. [143]	2017	20 females	Recreational runners	20 m running at 5.0 m/s
Liew et al. [110]	2021	10 males + 7 females	Healthy	45° cut at 4 m/s approach velocity
Lorimer et al. [53]	2018	12 males	Well-trained triathletes	2 min running on treadmill at 3.0, 3.3, 3.7, and 4.2 m/s
Lum et al. [129]	2019	14 males	Moderately trained endurance runners	10 km running on treadmill at 10 km/h and 12 km/h
Lussiana and Gindre [84]	2016	31 runners	Well-trained runners	15 min running at self-selected velocity
Lussiana et al. [85]	2017	58 males	Recreational runners	5 min running on treadmill at 12 km/h
Meur et al. [94]	2013	43 males + 36 females	Elite triathletes	Performance of each participant was examined during the running section of the World Triathlon Grand Final
Meyers et al. [67]	2019	375 boys	Biweekly physical education classes	30 m sprint
Meyers et al. [71]	2016	189 boys	Biweekly physical education classes	30 m sprint
Meyers et al. [72]	2017	344 boys	Biweekly physical education classes	35 m sprint
Monte et al. [65]	2017	20 males + 20 females	Elite and intermediate sprinters	80 m sprint with different stride frequencies (preferred and +15%, +30%, −15%, and −30% of the self-selected)
Monte et al. [68]	2020	32 males	Endurance runners	6 min running on treadmill at theoretical half-marathon running velocity
Morin et al. [139]	2005	8 + 10 males	Physical education students + elite middle − distance runners	Running on treadmill at 3.33, 3.89, 4.44, 5.0, 5.56, 6.11, and 6.67 m/s + 10 m running at 4.0, 5.0, 6.0, and 7.0 m/s and maximal velocity
Morin et al. [55]	2006	8 males	Physical education students	100 m sprint
Morin et al. [92]	2012	11 males	Physically active physical education students	Running on treadmill at 10 and 20 km/h
Nagahara and Zushi [127]	2017	9 males	Sprinter, 2 jumpers, 5 pole vaulters, and a decathlete	60 m sprint
Pappas et al. [147]	2014	22 males	Healthy physical education students	Running on treadmill at 4.44 m/s
Paradisis et al. [58]	2019	50 males	Subelite sprinters	35 m sprint
Powell et al. [168]	2017	20 females	Recreational athletes	Running at self-selected velocity
Rabita et al. [100]	2013	12 males	Runners	Running to exhaustion at constant velocity corresponding to VO_2max_
Rabita et al. [99]	2011	6 males + 3 females	Elite triathletes	Running to exhaustion at a velocity corresponding to 95% of the VO_2max_
Rogers et al. [86]	2017	11 males	Highly trained middle-distance runners	50 m sprint
Rumpf et al. [73]	2015	32 children	Physically active and trained a minimum of two times per week	30 m sprint on treadmill
Rumpf et al. [70]	2013	74 boys	Physically active	30 sprint on treadmill
Shih et al. [114]	2019	20 males + 20 females	Recreational runners	14 m running at 3.4 m/s
Sinclair et al. [145]	2015	14 males + 14 females	Recreational runners	Running at 4.0 m/s
Stafilidis and Arampatzis [90]	2007	10 male	Experienced sprinters	60 m sprint
Weir et al. [98]	2020	13 males	Recreational runners	Prolonged running on treadmill (2 × 21 min)
Williams III et al. [166]	2004	18 males + 22 females	Healthy	25 m running at 3.35 m/s
Yin et al. [109]	2020	78 males	Healthy amateur runners	15 m running at 3.3 m/s

**Table 2:** List of the studies on vertical stiffness during running.

Authors	Year	Number of participants	Sport background	Motor skill
Ache-Dias et al. [128]	2018	18 (males + females)	Recreational runners	Submaximal constant load running test on treadmill (6 min at 9 km/h)
Arampatzis et al. [62]	1999	13 runners	Not mentioned	Running at 2.5, 3.5, 4.5, 5.5, and 6.5 m/s
Bitchell et al. [97]	2019	7 + 13 runners	Trained + untrained runners	Incremental running on treadmill
Brocherie et al. [81]	2015	8 males	International football players	RAST test (6 × 35 m sprint)
Cavagna et al. [60]	1988	10 males	Untrained	Running at a variety of different constant velocities (range of very low velocities)
Cavagna et al. [63]	2005	4 males + 1 female	Not mentioned	Running at different velocities (from 5.2 to 20.5 km/h)
Cherif et al. [77]	2017	21 males	Healthy and active	5 × 5 s sprints on treadmill
Choukou et al. [106]	2012	8 males	Sprinters competing at the regional level	100 m sprint
Cronin and Rumpf [69]	2014	16 males	Young athletes	30 m sprint on treadmill
Dal Pupo et al. [107]	2017	21 males	Futsal players	10 m sprint
Dalleau et al. [74]	1998	8 males	Healthy	Running on treadmill (4 min at a velocity corresponding to 90% of the VO_2max_)
Dutto and Smith [76]	2002	11 males + 4 females	Well-trained runners	Running on treadmill to exhaustion at a velocity corresponding to 80% of the VO_2max_
Farley and González [33]	1996	4 males	Experienced treadmill runners	Running on treadmill at 2.5 m/s (while using a range of stride frequencies from 26% below to 36% above the preferred stride frequency)
Ferris et al. [88]	1999	6 females	Healthy	17 m running at 3.0 m/s
Ferris et al. [87]	1998	5 humans	Not mentioned	Running at 5 m/s
Fourchet et al. [102]	2015	11 males	Highly trained middle-distance runners	Running on treadmill to exhaustion at a velocity corresponding to 95% of the VO_2max_
García-Pinillos et al. [103]	2020	22 males	Endurance runners	60 min running on treadmill
García-Pinillos et al. [66]	2019	22 males	Novice and elite endurance runners	Incremental running on treadmill at 10, 12, 14, 16, and 18 km/h
Gindre et al. [83]	2016	77 males + 14 females	Healthy and active	50 m running at 3.3, 4.2, and 5.0 m/s
Giovanelli et al. [172]	2017	12 males	Ultraendurance runners	6 h running “6 ore Città di Buttrio”
Giovanelli et al. [95]	2016	18 males	Ultraendurance runners	“Supermaratona dell'Etna”
Girard et al. [150]	2015	13 males	Team and racket sport background	3 × 5 s sprints on treadmill
Girard et al. [80]	2017	20 males	Field hockey players	6 × 30 s running on treadmill at 115% of the VO_2max_
Girard et al. [57]	2017	14 males	Recreationally intermittent sports	3 × 5 s sprints on treadmill + running on treadmill at 10 and 20 km/h
Girard et al. [56]	2016	11 males	Physical education students practicing a field sport	100, 200, and 400 m sprint on treadmill
Girard et al. [79]	2011	16 males	Recreational team or racket sports athletes	12 × 40 m sprints
Girard et al. [96]	2017	18 males	Physical education students	800 m running
Girard et al. [91]	2010	12 triathletes	Highly and well-trained triathletes	5000 m running at self-selected velocity
Girard et al. [93]	2013	12 males	National level triathletes	5000 m running at self-selected velocity
Girard et al. [78]	2011	13 males	Young soccer players	6 × 20 m sprints
Hayes and Caplan [101]	2014	6 runners	Subelite middle-distance runners	Running on treadmill to exhaustion at velocity corresponding to VO_2max_
He et al. [61]	1991	4 males	Healthy	Running on treadmill at 2.0, 3.0, 4.0, 5.0, and 6.0 m/s
Heise and Martin [75]	1998	16 males	Recreational runners	15 m running at 3.35 m/s
Hobara et al. [64]	2010	8 males	Well-trained sprinters and runners	400 m sprint
Hunter [157]	2003	9 males + 7 females	Not mentioned	10 min running on treadmill at self-selected velocity
Hunter and Smith [105]	2007	11 males + 5 females	Recreational runners	1 h running on treadmill at constant velocity
Joseph et al. [148]	2013	20 males	Various sports	10 m running at 3.35 m/s
Joseph et al. [121]	2014	20 males	Various sports	10 m running at 3.35 m/s
Kuitunen et al. [59]	2002	10 males	Sprinters	Sprint at 70%, 80%, 90%, and maximal velocity
Lorimer et al. [53]	2018	12 males	Well-trained triathletes	2 min running on treadmill at 3.0, 3.3, 3.7, and 4.2 m/s
Lum et al. [129]	2019	14 males	Moderately trained endurance runners	10 km running on treadmill at 10 km/h and 12 km/h
Luhtanen and Komi [156]	1980	6 athletes	Track and field athletes	Running at 40%, 60%, 80%, and maximal velocity
Lussiana et al. [85]	2017	58 male	Recreational runners	5 min running on treadmill at 12 km/h
McMahon et al. [82]	1987	6 males	Healthy	30 m constant velocity running
Meur et al. [94]	2013	43 males + 36 females	Elite triathletes	Performance of each participant was examined during the running section of the World Triathlon Grand Final
Meyers et al. [67]	2019	375 boys	Biweekly physical education classes	30 m sprint
Meyers et al. [71]	2016	189 boys	Biweekly physical education classes	30 m sprint
Meyers et al. [72]	2017	344 boys	Biweekly physical education classes	35 m sprint
Monte et al. [65]	2017	20 males + 20 females	Elite and intermediate sprinters	80 m sprint with different stride frequencies (preferred and +15%, +30%, −15%, and −30% of the self-selected)
Monte et al. [68]	2020	32 males	Endurance runners	6 min running on treadmill at theoretical half-marathon running velocity
Morin et al. [139]	2005	8 + 10 males	Physical education students + elite middle − distance runners	Running on treadmill at 3.33, 3.89, 4.44, 5.0, 5.56, 6.11, and 6.67 m/s + 10 m running at 4.0, 5.0, 6.0, and 7.0 m/s and maximal velocity
Morin et al. [55]	2006	8 males	Physical education students	100 m sprint
Morin et al. [92]	2012	11 males	Physically active physical education students	Running on treadmill at 10 and 20 km/h
Nagahara and Zushi [127]	2017	9 males	Sprinter, 2 jumpers, 5 pole vaulters, and a decathlete	60 m sprint
Pappas et al. [147]	2014	22 males	Healthy physical education students	Running on treadmill at 4.44 m/s
Paradisis et al. [58]	2019	50 males	Subelite sprinters	35 m sprint
Rabita et al. [100]	2013	12 males	Runners	Running to exhaustion at constant velocity corresponding to VO_2max_
Rabita et al. [99]	2011	6 males + 3 females	Elite triathletes	Running to exhaustion at a velocity corresponding to 95% of the VO_2max_
Rogers et al. [86]	2017	11 males	Highly trained middle-distance runners	50 m sprint
Roschel et al. [130]	2015	15 humans	Recreational runners	Submaximal running tests on treadmill (10 min at 12 km/h and 90% ventilatory threshold intensity)
Rumpf et al. [73]	2015	32 children	Physically active and trained a minimum of two times per week	30 m sprint on treadmill
Rumpf et al. [70]	2013	74 boys	Physically active	30 sprint on treadmill
Stafilidis and Arampatzis [90]	2007	10 males	Experienced sprinters	60 m sprint
Vincent et al. [146]	2020	28 males + 26 females	Recreational runners	Running on treadmill at self-selected velocity
Yin et al. [109]	2020	78 males	Healthy amateur runners	15 m running at 3.3 m/s

**Table 3:** List of the studies on joint stiffness during running.

Authors	Year	Number of participants	Sport background	Motor skill	Stiffness measure
Aeles et al. [119]	2018	7 males + 9 females and 11 males + 10 females	Adult well − trained sprinters + well − trained young athletes	10 m sprint	Ankle joint
Arampatzis et al. [62]	1999	13 runners	Not mentioned	Running at 2.5, 3.5, 4.5, 5.5, and 6.5 m/s	Knee joint, ankle joint
Chan et al. [126]	2020	20 males	Recreational distance runners	Running on treadmill (30 min at self-reported velocity)	Knee joint, ankle joint
Charalambous et al. [120]	2012	1 male	Internationally competitive sprint hurdle athlete	Maximal sprint starts with 10 m acceleration	Ankle joint
Günther and Blickhan [122]	2002	8 males + 4 females	Sports students and active sportsmen	Running at convenience velocity (from 3.7 to 5.6 m/s)	Knee joint, ankle joint
Hamill et al. [125]	2014	27 males + 13 females	Runners	25 m running at 3.5 m/s	Knee joint, ankle joint
Hamill et al. [112]	2009	33 runners	Runners	Running on treadmill at 3.8 m/s	Hip joint, knee joint, ankle joint
Jin and Hahn [113]	2018	5 males + 5 females	Healthy	Running on treadmill (from 1.8 to 3.8 m/s)	Hip joint, knee joint, ankle joint
Joseph et al. [148]	2013	20 males	Various sports	10 m running at 3.35 m/s	Knee joint, ankle joint
Kuitunen et al. [59]	2002	10 males	Sprinters	Sprint at 70%, 80%, and 90% and maximal velocity	Knee joint, ankle joint
Lorimer et al. [53]	2018	12 males	Well-trained triathletes	2 min running on treadmill at 3.0, 3.3, 3.7, and 4.2 m/s	Hip joint, knee joint, ankle joint
Mager et al. [118]	2018	11 males + 16 females	Healthy students	Running at self-selected velocity	Ankle joint
Melcher et al. [124]	2017	13 males	Well-trained runners	25 m running with a 15 m acceleration	Knee joint, ankle joint
Nagahara and Zushi [127]	2017	9 males	Sprinter, 2 jumpers, 5 pole vaulters, and a decathlete	60 m sprint	Knee joint, ankle joint
Powell et al. [167]	2014	20 females	Recreational athletes	Running at self-selected velocity	Ankle joint
Shih et al. [114]	2019	20 males + 20 females	Recreational runners	14 m running at 3.4 m/s	Hip joint, knee joint, ankle joint
Sinclair et al. [145]	2015	14 males + 14 females	Recreational runners	Running at 4.0 m/s	Knee joint, ankle joint
Stefanyshyn and Nigg [117]	1998	10 males	Distance runners and sprinters	Running at 4 m/s and maximal acceleration sprint	Ankle joint
Tam et al. [115]	2017	14 males	Elite runners	60 m running at 12 and 20 km/h	Knee joint, ankle joint
Tam et al. [123]	2019	30 males	Runners	60 m running at 3.3 m/s	Knee joint, ankle joint
Verheul et al. [116]	2017	26 (males + females)	Runners	70 m running at 2.5, 3.5, 4.5, and 5.5 m/s and maximal velocity	Knee joint
Weir et al. [98]	2020	13 males	Recreational runners	Prolonged running on treadmill (2 × 21 min)	Knee joint, ankle joint
Williams III et al. [166]	2004	18 males + 22 females	Healthy	25 m running at 3.35 m/s	Knee joint

**Table 4:** List of the longitudinal studies on training effects on mechanical stiffness.

Authors	Year	Number of participants	Sport background	Motor skill	Stiffness measure
Ache-Dias et al. [128]	2018	18 (males + females)	Recreational runners	Submaximal constant load running test on treadmill (6 min at 9 km/h)	Leg, vertical
Lum et al. [129]	2019	14 males	Moderately trained endurance runners	10 km running on treadmill at 10 km/h and 12 km/h	Leg, vertical
Nagahara and Zushi [127]	2017	9 males	Sprinter, 2 jumpers, 5 pole vaulters, and a decathlete	60 m sprint	Leg, vertical, knee joint, ankle joint
Roschel et al. [130]	2015	15 humans	Recreational runners	Submaximal running tests on treadmill (10 min at 12 km/h and 90% ventilatory threshold intensity)	Vertical
Rumpf et al. [73]	2015	32 children	Physically active and trained a minimum of two times per week	30 m sprint on treadmill	Leg, vertical
